This article has been retracted.

# Risk Factors Affecting the Infusion Rate of Chemotherapeutic Agents within 2 Hours after Preparation and the Intervention Effect of the Quality Control Circle

**DOI:** 10.1155/2022/1856075

**Published:** 2022-10-12

**Authors:** Xiao Wu, Xinxin Chen, Lihang He

**Affiliations:** Department of Pharmacy Department, Dongyang People's Hospital, Jinhua, 322100 Zhejiang, China

## Abstract

**Objective:**

To investigate the risk factors for the infusion rate of chemotherapeutic agents within 2 hours after preparation and to observe the application effect of the quality control circle.

**Methods:**

The infusion rates of chemotherapeutic agents within 2 hours after the preparation in different wards of our hospital in February 2019 were counted and relevant factors were collected. Binary logistic regression analysis was utilized to screen the risk factors for the infusion rate of chemotherapeutic agents within 2 hours after the preparation. In March 2019, the quality control circle intervention was implemented according to risk factors. The application effect of the quality control circle was observed.

**Results:**

Logistic regression analysis results exhibited that insufficient attention to key performance indicator (KPI), heavy workload, forgotten or unfamiliar KPI, no real-time attention by the head of the department, simultaneous preparation of multiple groups of infusions for the same patient, preparation of all chemotherapeutic agents in the morning, and self-prepared medicine without a medical order were independent risk factors for infusion of chemotherapeutic agents beyond 2 hours after preparation (*P* < 0.05). The infusion rate of the chemotherapeutic agents (96.54%) within 2 hours after the preparation was significantly higher after the application of the quality control circle than that before the application (60.45%). The improvement rate was 59.65% and the goal achievement rate was 104.37% (*P* < 0.01).

**Conclusion:**

Insufficient attention to KPI, heavy workload, forgotten or unfamiliar KPI, no real-time attention by the head of the department, simultaneous preparation of multiple groups of infusions for the same patient, preparation of all chemotherapeutic agents in the morning, and self-prepared medicine without a medical order are crucial risk factors for limiting the increase in the infusion rate of chemotherapeutic agents within 2 hours after the preparation. Quality control circle intervention based on risk factors can effectively improve the infusion rate of chemotherapeutic agents within 2 hours after the preparation.

## 1. Introduction

The basis for safe infusion and efficacy is to guarantee the safety and stability of drug compatibility. The stability and infusion time of finished products after medicine preparation in the Pharmacy Intravenous Admixture Services (PIVAS) are easily overlooked by clinicians [1]. A previous study has found that the stability and efficacy of antitumor drugs after compatibility are strongly associated with the storage environment and infusion time limit. Long storage time easily reduced drug efficacy and stability and caused adverse reactions [2]. Chemotherapeutic agents such as paclitaxel injection and homoharringtonine injection should be infused for more than 3 hours. Therefore, the infusion should be started within 2 hours at the latest after the preparation of chemotherapeutic agents to ensure the quality of finished products [3]. It is clearly stated in the relevant norms and guidelines that the prepared solution should not be placed for more than 2 hours [4, 5]. Nevertheless, the infusion rate of intravenous drugs, especially intravenous chemotherapeutic agents, is relatively low within 2 hours after preparation in the clinic. In previous clinical investigations, the infusion rate of chemotherapeutic agents within 2 hours after preparation was only approximately 60% in our hospital, which was far from meeting the requirements of the above-mentioned regulations. Taken together, clarifying the risk factors for the infusion rate of chemotherapeutic agents within 2 hours after the preparation and giving active interventions have positive effects on shortening the waiting time of the finished chemotherapeutic agents, improving the quality of chemotherapeutic agents during infusion, and ensuring the efficacy and medication safety. This study was designed to analyze the risk factors for the infusion rate of chemotherapeutic agents within 2 hours after the preparation and to observe the application effect of the quality control circle.

## 2. Data and Methods

### 2.1. General Information

Patients who received a chemotherapeutic agents in different wards of our hospital in February 2019 were recruited as subjects. A total of 536 intravenous chemotherapeutic agent preparations were made in 14 wards in February 2019. There were 170 males and 140 females, aged 29-90 years old, mean (59.71 ± 11.37) years old. Among 536 preparations, there were 201 cases in group 1, 56 cases in group 2, 36 cases in group 3, 4 cases in group 4, 3 cases in group 5, 1 case in group 6, 4 cases in group 7, 2 cases in group 8, 2 cases in group 10, and 1 case in group 14. The quality control circle intervention was implemented from March 2019 to March 2020, with February 2019 as the preapplication period and March 2020 as the postapplication period. All patients receiving chemotherapy drug infusion during this period were included in the study. Before and after the application of the quality control circle, the infusion rates of chemotherapeutic agents within 2 hours after the preparation were observed in different wards of our hospital.

### 2.2. Methods

#### 2.2.1. Risk Factor Analysis

The patients receiving chemotherapeutic agents in different wards of our hospital in February 2019 were enrolled as subjects. The infusion rates within 2 hours after the 536 preparations of intravenous chemotherapeutic agents were observed in 310 patients from the 14 wards in February 2019. Personnel, process, equipment, and other relevant factors were collected. Personnel factors include nursing staff [insufficient attention to key performance indicator (KPI)/heavy workload], delivery staff (delayed delivery/the medicine was delivered to the department without notifying the nurse), preparation staff (failure to leave the warehouse in time after the preparation/delayed preparation), new employees (forgotten or unfamiliar KPI/unfamiliar process), and the head of the department (no real-time attention). Process factors contain medical order request (scattered/late), preparation process (simultaneous preparation of multiple groups of infusions for the same patient/failure to leave the warehouse in time after preparation/preparation of all chemotherapeutic agents in the morning/late preparation), and package and delivery (delivery of prepared finished products and newly issued medical orders together/the medicine cannot be delivered by a medicine elevator, because it is not in the same building). Equipment factors consist of the slow drug dissolution speed of the oscillator, slow speed induced by the inflexibility of the medicine delivery vehicle, and long waiting time for the elevator. Other factors include special medicines (chemotherapy pump and long albumin-bound paclitaxel preparation time) and self-prepared medicines (many self-prepared medicines/late delivery of self-prepared medicines/self-prepared medicine without a medical order). Univariate analysis and logistic regression analysis were employed to observe the risk factors for the infusion rate of chemotherapeutic agents within 2 hours after the preparation.

#### 2.2.2. Quality Control Circle Intervention

Following risk factors, a quality control circle intervention was performed in March 2019. The details are as follows: (1) establishment. The quality control circle team was established with 7 members, and the average age was (33.71 ± 6.33) years. All of the members had bachelor's degree, with 2 pharmacists, 1 pharmacist in charge, 2 nurse in charge, 1 deputy chief pharmacist, and 1 engineer. The theme of the activity was “improving the infusion rate of chemotherapeutic agents within 2 hours after the preparation”. (2) Activity plan formulation. The activities were carried out from March 2019 to March 2020. From March to May, weekly theme selection, activity planning, status grasp, goal setting, analysis, countermeasure formulation, countermeasure implementation and self-criticism, effectiveness confirmation, standardization, self-criticism, and improvement were conducted. The period from June to March of the following year was the implementation stage of the plan, and April of the following year was the stage of achievement confirmation. (3) Grasping the current situation. After understanding the current dispensing and delivery of chemotherapeutic agents, the target was determined according to the screening factors, discussed, and analyzed to give targeted improvement countermeasures. (4) Goal setting. Taking the infusion rate of chemotherapeutic agents within 2 hours after the preparation in each ward of the hospital as a reference in February 2019, the goal was to increase the infusion rate within 2 hours after the preparation to 95% after quality control circle intervention. (5) Analysis. The fishbone diagram was utilized to analyze the correlation among various factors, and “1.2.1 Risk factor analysis” was applied to screen the main factors affecting the infusion rate of chemotherapeutic agents within 2 hours after the preparation and to formulate corresponding countermeasures. (6) Countermeasure formulation. For each evaluation item, all members could evaluate various countermeasures according to indicators such as feasibility, economy, and circle ability—the 80/20 principle is the implementation countermeasure. According to the similarity, the countermeasures were organized into countermeasure 1, “prepared in batches according to the order of clinical use”; countermeasure 2, “daily statistical inspection data and the statistical results were published in the head nurse's WeChat group every month”; and countermeasure 3, “self-prepared medicines are included in the homogeneous management of medical orders”. (7) Countermeasure implementation and self-criticism. (7.1) Preparation in batches according to the order: at this stage, chemotherapeutic agents were mostly prepared in the morning. The infusion interval was too long after preparation, which affected the efficacy and had potential security risks. Given this problem, the chemotherapeutic agents would be prepared in batches according to clinical needs. There were two batches in the morning and two batches in the afternoon. The doctor was coordinated to remark the batches when making the medical order. Pharmacy Intravenous Admixture Services arranged the warehousing according to the batches in the remarks. The first and second batches were prepared in the morning. The third and fourth batches were prepared in the afternoon. If the batch was not remarked or the batch needed to be changed, the nurse in the office would notify by phone. The standardization was conducted after the preliminary confirmation of the effect. The “Operation Instructions for the Dispensing and Delivery of Chemotherapeutic Agents” was formulated and studied by related people. (7.2) Data monitoring and verification: after studying KPI standards, the infusion rate of the previous day was counted every morning. The departments and patients who had been infused with overtime were paid attention to. The infusion time was checked. The batch was adjusted according to the situation on the day of the medical order. The inspection data of the previous month was counted at the beginning of each month. (7.3) Homogeneous management of self-prepared medicines: currently, self-prepared medicines did not have a catalog in the information system and they could only be remarked in the remark column of the solvent medical order. The medical order could not enter the Pharmacy Intravenous Admixture Services, and the self-prepared medical order could not be counted. Furthermore, the characters in the remark column on the label were limited; sometimes, the medicine name and dosage could not be displayed completely. In response to the above problems, departments that needed to use self-prepared medicines could apply for the self-prepared medicine list, which was added to the hospital HIS system with the approval of the purchasing center. When a doctor prescribed a medical order, self-prepared medicine would be automatically displayed and the word “self-prepared” would be displayed on the label of the medical order. (8) Effect confirmation. (8.1) Visible results: after the improvement, the infusion rate within 2 hours after the preparation increased to 96.51% and the goal achievement rate was 104.37%. (8.2) Intangible results: the members of the quality control circle team had improved in all aspects of enthusiasm, sense of honor, communication and cooperation, cohesion, problem-solving ability, and quality control techniques. (9) Standardization. A standard workbook has been formulated—the Operation Instructions for the Dispensing and Delivery of Chemotherapeutic Agents. (10) Self-criticism and improvement. (10.1) Clinicians would forget to remark batches, so infusion time exceeded 2 hours. (10.2) Sometimes, the pharmacy label could not match the infusion label, so the label scan before preparation was unsuccessful. The system did not have the preparation time, so the infusion rate statistics were affected. (10.3) The publicity and education on batch remarks of medical orders were carried out regularly. The problem of label mismatch was fed back to the information department and solved.

### 2.3. Observation Indicators and Definitions

(1) Infusion rate within 2 hours: *infusion* *rate* *within* 2 *hours* = *number* of *infusions* *within* 2 *hours*/*total* *number* of *preparations* of *chemotherapeutic* *agents* in the *current* *month* × 100%. The number of infusions within 2 hours is the number of infusions of chemotherapeutic agents from the preparation to the start of infusion in the ward, which is controlled within 2 hours. (2) Influencing factors: the factors affecting the infusion rate within 2 hours were determined by using univariate analysis and logistic multivariate analysis. (3) Improvement rate: with February 2019 as the preapplication period and March 2020 as the postapplication period, the quality control circle intervention was implemented in March 2019 to detect the infusion rate within 2 hours after the preparation of chemotherapeutic agents in various wards of our hospital. The data came from the infusion list in the preparation room. The time from preparation to the start of infusion was counted. Improvement rate and goal achievement rate were calculated as follows:*improvement* *rate* = (*infusion* *rate* *within* 2 *hours* *after* *improvement* − *infusion* *rate* *within* 2 *hours* *before* *improvement*)/*infusion* *rate* *within* 2 *hours* *before* *improvement* × 100%; *goal* *achievement* *rate* = (*data* *after* *improvement* − *data* *before* *improvement*)/(*goal* *value* − *data* *before* *improvement*) × 100%

### 2.4. Statistical Methods

All data were analyzed using SPSS 23.0 statistical software. Count data were expressed as cases (%) and analyzed utilizing the chi-square test. Kolmogorov-smirnov test was used to check whether the measurement data conform to normal distribution. Measurement data were presented as the mean ± standard deviation and analyzed using a *t*-test. Binary logistic regression analysis was applied to observe the risk factors for the infusion rate within 2 hours. A value of *P* < 0.05 was considered statistically significant.

## 3. Results

### 3.1. Infusion Rate within 2 Hours in each Department of our Hospital before the Application of the Quality Control Circle

In February 2019, 536 preparations of chemotherapeutic agents were observed in 310 patients undergoing chemotherapy from the 14 departments of our hospital. The number of infusions within 2 hours was 324 and the number of infusions beyond 2 hours was 212. The infusion rate within 2 hours was 60.45% (324/536). The infusion rates within 2 hours in different departments are displayed in Figure 1.

### 3.2. Univariate Analysis of the Infusion Rate within 2 Hours after Preparation of Chemotherapeutic Agents

The influential factors for the infusion rate within 2 hours after preparation of chemotherapeutic agents contained insufficient attention to KPI, heavy workload, delayed delivery, failure to leave the warehouse in time after the preparation, forgotten or unfamiliar KPI, unfamiliar process, no real-time attention by the head of the department, scattered medical order request, late medical order request, simultaneous preparation of multiple groups of infusions for the same patient, preparation of all chemotherapeutic agents in the morning, delivery of prepared finished products and newly issued medical orders together, inflexibility of the medicine delivery vehicle, many self-prepared medicines or late delivery of self-prepared medicines, and self-prepared medicine without a medical order (*P* < 0.05; Table 1).

### 3.3. Multivariate Analysis of the Infusion Rate within 2 Hours after Preparation of Chemotherapeutic Agents

The significant factors of univariate analysis were utilized as independent variables to be substituted into binary logistic regression analysis. The infusion time after preparation of chemotherapeutic agents was used as the dependent variable (infusion within 2 hours = 0, infusion beyond 2 hours = 1). Independent variable assignment: insufficient attention to KPI (yes = 1, no = 0), heavy workload (yes = 1, no = 0), delayed delivery (yes = 1, no = 0), failure to leave warehouse in time after preparation (yes = 1, no = 0), forgotten or unfamiliar KPI (yes = 1, no = 0), unfamiliar process (yes = 1, no = 0), no real-time attention by the head of the department (yes = 1, no = 0), scattered medical order request (yes = 1, no = 0), late medical order request (yes = 1, no = 0), simultaneous preparation of multiple groups of infusions for the same patient (yes = 1, no = 0), preparation of all chemotherapeutic agents in the morning (yes = 1, no = 0), delivery of prepared finished products and newly issued medical orders together (yes = 1, no = 0), inflexibility of the medicine delivery vehicle (yes = 1, no = 0), many self-prepared medicines or late delivery of self-prepared medicines (yes = 1, no = 0), and self-prepared medicine without a medical order (yes = 1, no = 0). Logistic regression analysis results exhibited insufficient attention to KPI, heavy workload, forgotten or unfamiliar KPI, no real-time attention by the head of the department, simultaneous preparation of multiple groups of infusions for the same patient, preparation of all chemotherapeutic agents in the morning, and self-prepared medicine without a medical order were independent risk factors for infusion beyond 2 hours after preparation of chemotherapeutic agents (*P* < 0.05; Table 2).

### 3.4. Application Effect of the Quality Control Circle

The evaluation results displayed that the infusion rate (96.54%) within 2 hours after the preparation of chemotherapeutic agents was significantly higher after the application of the quality control circle than that before the application (60.45%). The improvement rate was 59.65% and the goal achievement rate was 104.37% (*P* < 0.01; Table 3, Figure 2).

## 4. Discussion

The stability of chemotherapeutic agents after compatibility has always been the focus of clinical attention and is strongly associated with the occurrence of drug-related adverse reactions and the clinical application effect. The influence of time on the stability of medicines including chemotherapeutic agents after compatibility has been widely recognized. Due to the influence of various factors such as physical condition, disease, and clinical treatment, the physical tolerance is remarkably diminished, and the probability of drug-related adverse reactions during clinical treatment is dramatically increased in patients with malignant diseases. Prolonged placement time or long infusion time may aggravate the occurrence of adverse reactions and reduce efficacy. In other words, the time from the compatibility of chemotherapeutic agents to intravenous infusion may be an important factor affecting the efficacy and the occurrence of adverse reactions [6]. This conclusion has been confirmed in some previous studies. Zhang et al. [7] have concluded that drug preparation time is one of the high-risk factors for adverse reactions to intravenous infusion in children. A study by Chen has confirmed that the factors affecting the effect of chemotherapeutic agents mainly include solvents, dissolution method, and preparation time [8]. It can be seen that the preparation time of clinical drugs also plays an important role in ensuring clinical efficacy and diminishing adverse reactions.

Although nosocomial infection management standards in wards and nursing practice guidance and implementation rules for infusion therapy made clear instructions on the infusion time after preparation in the early years, heavy clinical work, lack of medical staff, lax individual work, and institutional management omissions seriously decrease the infusion rate within 2 hours after the preparation of chemotherapeutic agents [9]. A survey conducted in this study in February 2019 found that the infusion rate (60.45%) within 2 hours after the preparation of chemotherapeutic agents in various departments of the hospital was seriously lower than the infusion rate (95%) given by relevant regulations. The effect of preparation time on chemotherapeutic agents has gradually been paid attention to in the clinic. Strengthening the management after drug preparation has become an urgent problem to be solved at this stage. Due to the lack of relevant studies, the risk factors affecting the infusion of chemotherapeutic agents within 2 hours after preparation have not yet been identified. Therefore, this study sought to clarify the risk factors affecting the infusion of chemotherapeutic agents within 2 hours after preparation. According to the actual situation of our hospital, active improvement measures are given to improve the clinical work efficiency, enhance the infusion rate within 2 hours, and ensure clinical efficacy and medication safety.

This study enrolled patients undergoing intravenous chemotherapy in our hospital in February 2019 as subjects and observed the infusion rate within 2 hours after the preparation of chemotherapeutic agents in various departments. Univariate analysis results demonstrated that insufficient attention to KPI, heavy workload, delayed delivery, failure to leave the warehouse in time after the preparation, forgotten or unfamiliar KPI, unfamiliar process, no real-time attention by the head of the department, scattered medical order request, late medical order request, simultaneous preparation of multiple groups of infusions for the same patient, preparation of all chemotherapeutic agents in the morning, delivery of prepared finished products and newly issued medical orders together, inflexibility of the medicine delivery vehicle, many self-prepared medicines or late delivery of self-prepared medicines, and self-prepared medicine without a medical order were factors affecting the infusion rate within 2 hours after the preparation of chemotherapeutic agents (*P* < 0.05). KPI is a performance evaluation indicator widely used in medical institutions at present and has positive effects on improving hospital quality management and controlling hospital infection. KPI is also an important learning content for medical workers. Nevertheless, there are marked differences in the understanding and cognition of KPI among hospital workers. The heavy daily work inevitably causes clinical workers to have behaviors that are inconsistent with standards and norms [10]. Our logistic regression analysis results displayed that insufficient attention to KPI and forgotten or unfamiliar KPI were independent risk factors for the infusion beyond 2 hours after preparation (*P* < 0.05), suggesting that clinical attention should be paid to KPI learning and education to improve the behavioral norms of medical staff. In previous clinical work, most of the intravenous drugs in medical orders only have compatibility information but lack batch information, which leads to the concentrated preparation of many drugs and undoubtedly prolongs the shelving time of subsequent batches [11]. The logistic regression analysis results displayed that the simultaneous preparation of multiple groups of infusions for the same patient and preparation of all chemotherapeutic agents in the morning were independent risk factors for the infusion of chemotherapeutic drugs beyond 2 hours after preparation (*P* < 0.05), which was consistent with the above theory. In the previous work mode, the relevant data were counted and checked once a month under normal circumstances. Regarding the relevant normative requirements for the infusion of chemotherapeutic agents within 2 hours after preparation, not only the awareness rate of ordinary medical staff is low but also the heads of the departments have similar problems. The awareness rate and importance of the monthly statistical results are still low among the heads of various departments, and problems cannot be discovered and solved in time. The logistic regression analysis results demonstrated that no real-time attention by the head of the department was an independent risk factor for the infusion of chemotherapeutic agents beyond 2 hours after preparation (*P* < 0.05), reflecting that the head of the department plays an important role in supervision and management. The head's attention to this issue and the improvement of the existing work and study mode are not only conducive to improving the infusion rate within 2 hours after the preparation but also conducive to the study and mastery of the KPI for the staff in the department. Due to differences in hospital levels and regions, self-prepared medicine is a common problem in the treatment of malignant tumors at this stage. In the past, self-prepared medicines in the information system could only be remarked in the remark column of the solvent medical order, and the remarks were limited; self-prepared medicines have been neglected in the fast-paced work and the preparation was delayed [12]. The logistic regression analysis results showed that self-prepared medicine without a medical order is an independent risk factor for infusion of chemotherapeutic drugs beyond 2 hours after preparation (*P* < 0.05).

According to the data of this study, there are many factors affecting the infusion rate within 2 hours after the preparation of chemotherapeutic agents, but it is difficult to completely avoid them in the clinic. Therefore, key factors are selected to implement quality control circle intervention. Since the establishment of the quality control circle team in 2010, the quality control circle has been extensively used in the work of the pharmacy department of our hospital and has exerted a crucial effect on improving the operation process of the pharmacy department, improving work performance, and ensuring the safety of patients' medication [13]. According to the key risk factors, activities were carried out from March 2019 to March 2020 to improve the infusion rate within 2 hours after preparation. Our results concluded that the infusion rate (96.54%) within 2 hours after the preparation of the chemotherapy drugs was significantly higher after the application than that before the application of the quality control circle (60.45%). The improvement rate was 59.65% and the goal achievement rate was 104.37% (*P* < 0.01).

In summary, insufficient attention to KPI, heavy workload, forgotten or unfamiliar KPI, no real-time attention by the head of the department, simultaneous preparation of multiple groups of infusions for the same patient, preparation of all chemotherapeutic agents in the morning, and self-prepared medicine without a medical order are key risk factors limiting the increase in the infusion rate within 2 hours after preparation of chemotherapeutic agents. Quality control circle intervention based on risk factors can effectively improve the infusion rate within 2 hours after preparation.

## Figures and Tables

**Figure 1:** Histogram of the infusion rate within 2 hours after the preparation of chemotherapeutic agents in 14 departments of our hospital in February 2019.

**Figure 2:** Histogram of the infusion rate within 2 hours after the preparation of chemotherapeutic agents in each ward before and after the application of the quality control circle.

**Table 1:** Univariate analysis of infusion rate within 2 hours after the formulation of chemotherapeutic agents (*n* (%)).

Factors			Sum	Infusion within 2 h (*n* = 324)	Infusion beyond 2 h (*n* = 212)	*χ*2	*P*
Personnel factors	Insufficient attention to KPI	Yes	35	10 (28.57)	25 (71.43)	15.914	<0.001
		No	501	314 (62.67)	187 (37.33)		
	Heavy workload	Yes	21	8 (38.10)	13 (61.90)	4.567	0.032
		No	515	316 (61.36)	199 (38.64)		
	Delayed delivery	Yes	19	7 (36.84)	12 (63.16)	4.591	0.032
		No	517	317 (61.32)	200 (38.68)		
	Delivery to the department without notifying the nurse	Yes	21	9 (42.86)	12 (57.14)	2.829	0.092
		No	515	315 (61.17)	200 (38.83)		
	Failure to leave the warehouse in time after preparation	Yes	21	10 (47.62)	11 (52.38)	1.504	0.220
		No	515	314 (60.97)	201 (39.03)		
	Forgotten or unfamiliar KPI	Yes	21	8 (38.10)	13 (61.90)	4.567	0.032
		No	515	316 (61.36)	199 (38.64)		
	Unfamiliar process	Yes	23	9 (39.13)	14 (60.87)	4.567	0.032
		No	513	315 (61.40)	198 (38.60)		
	No real-time attention by the head of the department	Yes	26	9 (34.62)	17 (65.38)	7.627	0.005
		No	510	315 (61.76)	195 (38.24)		
Process factors	Scattered medical order request	Yes	23	9 (39.13)	14 (60.87)	4.567	0.032
		No	513	315 (61.40)	198 (38.60)		
	Late medical order request	Yes	26	10 (38.46)	16 (61.54)	5.525	0.018
		No	510	314 (61.57)	196 (38.43)		
	Simultaneous preparation of multiple groups of infusions for the same patient	Yes	24	8 (33.33)	16 (66.67)	7.726	0.005
		No	512	316 (61.72)	196 (38.28)		
	Failure to leave the warehouse in time after the preparation	Yes	25	10 (40.00)	15 (60.00)	4.586	0.032
		No	511	314 (61.45)	197 (38.55)		
	Preparation of all chemotherapeutic agents in the morning	Yes	29	10 (34.48)	19 (65.52)	8.645	0.003
		No	507	314 (61.93)	193 (38.07)		
	Late preparation	Yes	19	8 (42.11)	11 (57.89)	2.772	0.096
		No	517	316 (61.12)	201 (38.88)		
	Delivery of prepared finished products and newly issued medical orders together	Yes	27	11 (40.74)	16 (59.26)	4.619	0.031
		No	509	313 (61.49)	196 (38.51)		
	No direct delivery by the medicine elevator	Yes	20	9 (45.00)	11 (55.00)	2.074	0.149
		No	516	315 (61.05)	201 (38.95)		
Equipment factors	Slow drug dissolution speed	Yes	27	12 (44.44)	15 (55.56)	3.046	0.081
		No	509	312 (61.30)	197 (38.70)		
	Inflexibility of the medicine delivery vehicle	Yes	34	15 (44.12)	19 (55.88)	4.049	0.044
		No	502	309 (61.55)	193 (38.45)		
	Long waiting time for the elevator	Yes	26	14 (53.85)	12 (46.15)	0.498	0.480
		No	510	310 (60.78)	200 (39.22)		
Others	Chemotherapy pump, long albumin-bound paclitaxel preparation time	Yes	23	10 (43.48)	13 (56.52)	2.894	0.088
		No	513	314 (61.21)	199 (38.79)		
	Many self-prepared medicines or late delivery of self-prepared medicines	Yes	23	9 (39.13)	14 (60.87)	4.567	0.032
		No	513	315 (61.40)	198 (38.60)		
	Self-prepared medicine without a medical order	Yes	23	2 (8.70)	21 (91.30)	26.920	<0.001
		No	513	322 (62.77)	191 (37.23)		

**Table 2:** Logistic regression analysis of infusion rate within 2 hours after preparation of chemotherapeutic agents.

Factors	Regression coefficients	Standard error	Wald chi-square value	Significance	Exp (B)	95% confidence interval	
						Lower limit	Upper limit
Insufficient attention to KPI	1.259	0.419	9.032	0.003	3.523	1.550	8.011
Heavy workload	1.020	0.495	4.245	0.039	2.773	1.051	7.317
Delayed delivery	0.853	0.524	2.653	0.103	2.347	0.841	6.552
Failure to leave the warehouse in time after preparation	0.383	0.509	0.568	0.451	1.467	0.541	3.977
Forgotten or unfamiliar KPI	1.135	0.482	5.541	0.019	3.111	1.209	8.005
Unfamiliar process	0.909	0.488	3.471	0.062	2.482	0.954	6.457
No real-time attention by the head of the department	1.238	0.451	7.523	0.006	3.449	1.424	8.353
Scattered medical order request	0.937	0.479	3.824	0.051	2.553	0.998	6.529
Late medical order request	0.792	0.453	3.063	0.080	2.209	0.909	5.365
Simultaneous preparation of multiple groups of infusions for the same patient	1.352	0.468	8.334	0.004	3.866	1.544	9.680
Preparation of all chemotherapeutic agents in the morning	1.176	0.430	7.465	0.006	3.241	1.394	7.532
Delivery of prepared finished products and newly issued medical orders together	0.682	0.441	2.387	0.122	1.977	0.833	4.694
Inflexibility of the medicine delivery vehicle	0.624	0.398	2.456	0.117	1.867	0.855	4.074
Many self-prepared medicines or late delivery of self-prepared medicines	0.878	0.488	3.245	0.072	2.407	0.926	6.258
Self-prepared medicine without a medical order	2.526	0.776	10.582	0.001	12.501	2.729	57.263

**Table 3:** Comparison of the infusion rate within 2 hours after preparation of chemotherapeutic agents before and after the application of the quality control circle.

Time	Total number of times	Infusion within 2 h (times)	Infusion beyond 2 h (times)	Infusion rate within 2 h (%)	Improvement rate (%)	Goal achievement rate (%)
Before application (February 2019)	536	324	212	60.45	—	—
After application (March 2020)	1155	1115	40	96.54^∗^	59.65	104.37

Note: ^∗^*P* < 0.01 vs. before application.

## Data Availability

The simulation experiment data used to support the findings of this study are available from the corresponding authors upon request.
